# Leveled Design of Cryptography Algorithms Using Cybernetic Methods for Using in Telemedicine Applications

**DOI:** 10.1155/2021/3583275

**Published:** 2021-09-10

**Authors:** Ali Mohammad Norouzzadeh Gil Molk, Mohammad Reza Aref, Reza Ramazani Khorshiddoust

**Affiliations:** ^1^Department of Computer Engineering, Islamic Azad University, North Tehran Branch, Tehran, Iran; ^2^Department of Electrical Engineering, Sharif University of Technology, Tehran, Iran; ^3^Department of Industrial Engineering & Management Systems, Amirkabir University of Technology, Tehran, Iran

## Abstract

The technology world is developing fast with the developments made in the hardware and software areas. Considering that privacy and security of telemedicine applications are among the main necessities of this industry, as a result, there is a need to use lightweight and practical algorithms to be used in applications in the field of telemedicine, while security have the least negative impact. The distinct and contradicting components in the design and implementation of the cryptography algorithm, to achieve various objectives in medicine-based applications, have made it a complicated system. It is natural that, without identifying the components, indices, and properties of each system component, the hardware and software resources are lost and a proper algorithm cannot be designed. Accordingly, this paper presents a leveled model of cryptography algorithms using the cybernetic method. First, the main objectives and measures in the design of the cryptography algorithms are extracted using the measure reduction methods, and some of the excess and overlapping measures are eliminated. Then, three general classes of the cryptography algorithm design and implementation measures, applications of cryptography algorithms, and cryptography implementation techniques are extracted. Since the complexity of the cryptography algorithm design is relatively high, the cybernetic methodology is used to present a supermodel to make the cryptography algorithm design objective. Such design prevents examining unnecessary details and establishes a bidirectional relationship between the main design and implementation process and the support process. This relationship provides the support requirements of the main process by the support process at each step. Finally, the *Q*-analysis tools are used to analyse the proposed method, and the efficiency results are represented.

## 1. Introduction

Since telemedicine technology relies on data transmission, data security is critical in order to keep information transmission confidential and patients' privacy, and any potential threat or attack on telemedicine networks such as unauthorized access to data and alteration or destruction of patient data should be considered. In other words, any weakness in any part of the telemedicine network can affect the entire system. Therefore, in order to create security in the field of storage and exchange of information in the medical network, enforcement mechanisms using relevant standards should be considered. Accordingly, this study has focused on the surface design of cryptographic algorithms for use in telemedicine. Security of cryptography systems depends on “algorithm power” and “key size,” [1] and the general cryptography levels are divided into three levels, including cryptography algorithms, security protocols, and applications [2, 3]. However, the cryptography algorithms are designed and implemented to achieve goals such as confidentiality, authentication, and integrity [4], but various components such as speed, resource consumption, application type, flexibility, scalability, and reliability should be considered for their design. Design of a cryptography algorithm should be systematic, comprehensive, and staged. All required components of the information security should be considered in an excellence pattern in terms of technical, organization, procedural, and humanitarian aspects. Identifying new cryptographic challenges such as post-quantum cryptography and its agility, mobile applications, robustness of algorithms, and the role of implementation methods to achieve the above goals can be implemented in a comprehensive model [5–7]. Providing all these requirements simultaneously in the design of an algorithm is difficult and sometimes impossible. If contradictory objectives are considered for formulation of an objective/objectives of an algorithm, most algorithms might be broken, and if attacker has sufficient time, motivation, and resources, he can track the information [8]. Accordingly, presenting a model to make the cryptography algorithm design targeted is very important. Therefore, in this study, an approach is presented to design a leveled model of cryptography algorithms using the cybernetic method. The rest of this paper is structured as follows. In the second section, the literatures review is presented. In the third section, the cybernetic methodology is described, and a model is specified for design and implementation of cryptography algorithms based on extracted indices. In the fourth section, the proposed model is used to examine the design of the cryptography algorithm using the cybernetic supermodel. Finally, the proposed approach is evaluated using the *Q*-analysis method.

## 2. Literature Review

In [9], a security approach based on cryptography has been presented through examining the security issues in mobile devices and the available solutions. Also, it is mentioned that asymmetric cryptography is not a proper option for securing the resource-limited infrastructures such as IoT due to high complexity of the design and implementation. On the contrary, employing symmetric algorithms has other security issues. Accordingly, it has studied the design of cryptography algorithms based on position. To this end, an approach based on the AES algorithm and position of an efficient cryptography approach has been designed. In this approach, the application diagram is described and the user operation is studied. In the following, the operation flows of the system are described. Finally, it was evaluated that security can be increased through employing this approach. In [10], the design of stream cipher algorithms has been studied. It has been mentioned that stream cipher is one of the essential branches of symmetric cryptography, which requires limited hardware resources for execution. Therefore, considering the development of the communication technologies, the need to these algorithms is increasing. Accordingly, in the following, the design procedures and performance of various encryption algorithms, including NFSR, eStram, FCSR, and Panama, are presented through describing the main requirements of the cryptography algorithm design. The main purpose of this study is to present a perspective of stream cipher algorithm design and their performance. In 2016, NIST published a document called cipher standard and development instructions [11]. Transparency, openness, balance, accuracy, technical merit, global acceptability, usability, continuous improvement, and innovation and intellectual property (IIP) are the guidance principles of NIST cipher standards and development procedures. Also, NIST has started a procedure to request, evaluate, and standard of one or multiple public key cipher algorithms robust against quantum attacks [12]. In [11], lifecycle management processes and policies of cipher standard have been presented, where its main principles include: identifying and evaluating the needs, announcing the user's intention on a standard or instruction, considering the requirements and solutions, defining a specific program and procedure and design and development of a standard, and evaluating and maintaining the standard. In [13], an analytical framework has been presented to hardware and software implementation using cipher programs that verifies an integrated statistical framework which can implement the classified algorithms successfully based on a combination of heterogeneous hardware features and their software applications. The model presented in this paper includes six elements of goal, input, activities, output, outcomes, and performance. In [14], software engineering methodologies have been used to propose an adaptive approach for presenting a robust cipher key generation algorithm. The technique used in this method is based on self-checking procedures that can detect the system-level errors. Therefore, it can be used to check the security keys generated via employing random factors. These factors have been presented in the NIST evaluation results. In this software method, the values of the random factors are smaller than the acceptance values, and the key is generated when a valid value is detected. The generated keys are generated through shift register and SIGBA technique. The evaluation results indicate the efficiency of the presented approach in generating valid cipher keys. In [15, 16], security issues of mobile devices and processing infrastructure, including mobile computing and edge computing, have been studied. It has been concluded the importance of cipher algorithms and necessity of employing new models consider the complexity of these infrastructures. Bhowmik et al. [17] focused on security issues in telemedicine and introduced a double-tier (nDTCS) encryption system. Accordingly, this solution has proposed a modified logistic map and a congruence-based security model to secure telemedicine medical transactions. Two keys have been used for the encryption and decryption process, intermediate key and session key. The results of the evaluation indicate the effectiveness of the solution in order to secure the information through the proposing method [18]. In order to protect telemedicine communications, a key exchange solution is proposed by improving the Diffie–Hellman cryptographic algorithm. In this method, a randomized key generation is used to generate the key. The proposed solution is naturally safe and reliable due to the use of the Diffie–Hellman algorithm, so there is no need for recalculations or key reversal. The results of the evaluation also indicate that the proposed method is safe against guessing key attacks. In [19], an intelligent and secured transmission security solution for heart disease reports based on session key-based methods is presented. For this purpose, matrix confusion operations are used. The innovation of this solution is in the process of matrix transfer, which is transmitted in the form of a number of cardiologists in particular. Finally, the efficiency of the proposed method is evaluated with regard to cryptographic engineering, transparency, and strength. The results indicate that this method provides more security in the medical data transmission process. Hosseinian et al. [20] examined the importance of information security needs in telemedicine technology in the field of information transmission. In this study, the data collection tool was a questionnaire that was designed based on the criteria of the Association of Information Management and Health Care Systems (HMISS) in the field of telemedicine network security and security standards of the American Telemedicine Association. This questionnaire has been calculated separately based on a score of 1 to 5.  Table 1 summarizes the importance of each section.

## 3. Cybernetic Supermodel

Considering the complexity of the cipher context in terms of various aspects, designing a cipher algorithm should be systematic, comprehensive, and stage. To design cipher algorithms, different technologies, including mathematics, physics, biometric, biology, and social engineering, are used [21, 22]. Also, concepts and basic sciences such as theory of numbers, Boolean functions [23], and random functions [24, 25] are very essential. Depending of the application of cipher algorithms, various technical and nontechnical requirements should be considered for their design. Detecting new cryptography challenges such as postquantum cipher and its agility [26] and mobile applications [6, 7], making an algorithm robust, and the role of implementation methods to achieve the above goals are the issues that should be considered in a comprehensive model. Amidst, considering the large number of components in the design of cipher algorithms and their relationship and impact on each other, the design and implementation of these algorithms has become complicated. One of the best tools to design a complicated system is to present a model for that system. The steps associated with the design and implementation procedure of the cipher algorithm regardless of the triple classification of the hash, symmetric, and asymmetric functions at the highest level are shown in Figure 1.

Cryptography is one of the main information security components to transmit information from the sender to the receiver using the most secure method [27]. Design of the algorithms has different requirements depending on its application in the embedded or nonembedded system [28]. To design a robust algorithm, various technical and nontechnical factors should be considered so that the designed algorithm has sufficient robustness [29]. On the contrary, the effective factors should be in a coherent model with logical integration so that their impact on each other can be measured and evaluated; for instance, in [30–33], various algorithms have been evaluated in terms of some parameters. In fact, designing a conceptual model for the cipher algorithm requires considering all factors, components, and indices that affect the design and implementation of the cipher algorithms. Accordingly, in the design of the cipher algorithm, there should be a balance between “efficiency” and “resources” required for a specific security level [34]. Considering the design and generation process of the cipher algorithm and classification of factors, components, and indices, the conceptual cybernetic supermodel is used for design and implementation. Cybernetic is mainly focused on system performance and how they control their activities and communicate with their components. Therefore, the cybernetic pattern might be a scientific basis for making the cipher algorithms targeted. The cybernetic model of the cipher algorithms has four components of approach/strategy, main process, support process, and control process. The interactions of the main and support processes constitute the structure of the cipher system. These interactions result in a complicated diagram. To overcome this complexity, a leveled structure and mathematical facilities such as graph and matrix are used. Accordingly, the general cybernetic model for the design and implementation of the cipher algorithms is shown in Figure 2. This model is comprised of four sections: development approach/strategy process, main process, support process, and control process. The main process includes cryptography algorithms. The support process is divided into two general classes of hardware and software. The control process includes controlling the design, implementation, and controlling the outcome. As mentioned, this model is designed in the general level; and, its processes and components are studied in detail in Section 3.

Since the cipher algorithms have specific complexities, the component model is used to facilitate the processes. This type of design prevents spending time on unnecessary details. The strategic model for design of cipher algorithms should be presented at a level of detail that creates a trade-odd between “inclusion” and “applicability.” “Inclusion” indicated including various cipher algorithms. Accordingly, considering the component extracted for the main, support, and control section, a cybernetic model can be used to design and implement cipher algorithms in three levels, as shown in Figure 3. According to this model, there is a bidirectional relationship between the main design and implementation process and the support process; at each step, as a result of this relationship, the support requirements are demanded by the main process and provided by the support process.

### 3.1. Data Matrix of the Design Model Components

Since there are a large number of extracted objectives or measures in the design of cipher algorithms and some of them overlap, or eliminating some of them causes no problem for achieving the main goals, the criterion reduction method can be used to eliminate some measures. Accordingly, in this study, the approach presented in [19] is used to reduce the number of measures. In the feature reduction process, if eliminating one measure does not change the effective set of the problem, it is unnecessary. Therefore, after feature reduction, the component extraction process is carried out. In this step, three general classes of measures are extracted, including design and implementation objectives of cipher algorithms, applications of cipher algorithms, and implementation methods of the cipher algorithms. In the following, the reduced measures are classified into the above classes and modeling is carried out based on available measures of these three classes. Accordingly, based on the level-3 cybernetic model (Figure 3), the following three matrices are constituted to design and implement the cipher algorithms:

- The relationship matrix of support indices with main design and implementation processes of the cipher algorithms: since there are 13 support indices in the level-3 model (Figure 3) and 4 steps in the level-1 model (Figure 2), a 13∗4 matrix is constituted to determine the relationship between the members of these two processes, where its rows are the elements of the support process and its columns are the quadruple elements of the design and implementation of cryptography algorithms. The elements of this matrix are between 0 and 10, as shown in Table 2 [35]. The value of each element represents the effectiveness of each support index on each design and implementation step. Analysis of this matrix and its modeling computation provides the possibility for the policy-makers and developers to manage the resources required for each step of design and implementation of the cryptography algorithms and use the available hardware and software resources optimally.
- The relationship matrix of the objectives with the main design process of the cryptography algorithms: considering the seven objectives extracted in Section 2 and four steps in the main process, to determine the role of each step in achieving the seven objectives, a 7∗4 matrix is constituted. Since the number of final resources used to extract data is 814 papers, technical reports, and documents, the elements of this matrix are between 0 and 814, as given in Table 2. In this matrix, the value of each element represents the number of studies, documents, and reports indicating the relationship between two components. An interesting point in this matrix is that all algorithms implemented in the studied documents are evaluated.
- The relationship matrix of the implementation techniques and the design objectives of the cryptography algorithms: considering the 29 extracted techniques for cryptography algorithm implementation and seven main objectives of the cryptography algorithms, a 29 ∗ 7 matrix is constituted to determine how much each technique is used for cryptography implementation to achieve each objective (Table 3). The elements of this matrix are between 0 and 814. A part of this matrix is shown in Table 4.

#### 3.1.1. Design of Cryptography Algorithms Using the Cybernetic Supermodel

Considering the above discussion and presence of numerous indices and components in the design and implementation of the cryptography algorithm, which make it a complex system, identifying the relationship between these indices and ranking them is a necessity. Accordingly, in this section, the *Q*-analysis method is used and the output of the three matrices is analyzed. According to the level three of the proposed cybernetic model, the design and implementation support process of the cryptography algorithms includes 13 components. On the contrary, the design and implementation steps of the cryptography algorithms also include four steps, constituting a 13 ∗ 4 matrix.

### 3.2. Calculating the Incidence Matrix

First, the incidence matric is obtained based on the data matrix 4–1. This matrix represents the “impact of support indices on the main design process of the cryptography algorithms.” The data matrix is comprised of two sets *D*, support indices, set C, and quadruple design and implementation steps (Table 5). The incidence matrix calculated using the data matrix for *α*=%70 is represented in Table 6. By assigning different values to the parameter **α**, difference incidence matrices are obtained. The results of the *Q*-analysis using *C*++ coding for *α*=%70 are given in Figure 4:

(1) $$\begin{array}{c} D=\left\{d_{1},\;d_{2},\;\ldots ,\;d_{13}\right\},\\ C=\left\{c_{1},\;c_{2},\;c_{3},\;c_{4}\right\}. \end{array}$$

#### 3.2.1. Geometric Representation

Multidimensional properties of the system are defined by a simple or complex set *K*_*D*_(*C*, *λ*), such that the entities of the set *D* represent the support indices and entities of the set *C* represent the quadruple design and implementation steps of the cryptography algorithms.

In the sample with *α*_%70_=7, d_i_s is as follows:

(2) $$\begin{array}{c} d_{1}=\left\{\;\right\},\\ d_{2}=\left\{c_{1},\;c_{2},\;c_{3},\;c_{4}\right\},\\ d_{3\;}=\left\{c_{4}\right\},\\ d_{4\;}=\left\{c_{1},\;c_{3}\right\},\\ d_{5\;}=\left\{c_{1},\;c_{2},\;c_{3},\;c_{4}\right\},\\ d_{6\;}=\left\{c_{1},\;c_{2},\;c_{3},\;c_{4}\right\},\\ d_{7\;}=\left\{c_{1},\;c_{4}\right\},\\ d_{8\;}=\left\{c_{1},\;c_{2},\;c_{3},\;c_{4}\right\},\\ d_{9\;}=\left\{c_{1},\;c_{3},\;c_{4}\right\},\\ d_{10\;}=\left\{c_{1},\;c_{3},\;c_{4}\right\},\\ d_{11\;}=\left\{c_{1},\;c_{3},\;c_{4}\right\},\\ d_{12\;}=\left\{c_{1},c_{4}\right\}. \end{array}$$

The simplexes of *σ*_**p**_(**d**_**i**_) are also

(3) $$\begin{array}{c} \begin{array}{ccccccc} \sigma_{-1}\left(d_{1}\right) & \sigma_{3}\left(d_{2}\right) & \sigma_{0}\left(d_{3}\right) & \sigma_{1}\left(d_{4}\right) & \sigma_{3}\left(d_{5}\right) & \sigma_{0}\left(d_{3}\right) & \sigma_{1}\left(d_{7}\right)\\ \sigma_{3}\left(d_{8}\right) & \sigma_{2}\left(d_{9}\right) & \sigma_{2}\left(d_{10}\right) & \sigma_{2}\left(d_{11}\right) & \sigma_{1}\left(d_{12}\right) & \sigma_{1}\left(d_{13}\right) & \; \end{array}. \end{array}$$

Therefore, the complex dimension is 3. In other words, the diagnosis classes *d*_2_ (structure/organization), *d*_5_ (human resources/education), *d*_6_ (research and development), and *d*_8_ (management) have the largest dimension.

### 3.3. Calculating Dimensions and *Q*-Link

*Q*-link is defined as the link between a subset with smallest interface between two subsequent *d*_*i*_*s* in the chain of *d*_1_ to *d*_*n*_. *Q*-link between two subsequent *d*_i_*s* with **α**_%70_=7 is

(4) $$\begin{array}{c} \sigma_{-1}\left(d_{1}\right),\sigma_{3}\left(d_{2}\right)⟶1,\;\sigma_{3}\left(d_{2}\right),\sigma_{0}\left(d_{3}\right)⟶0,\sigma_{0}\left(d_{3}\right),\sigma_{1}\left(d_{4}\right)⟶-1,\\ \sigma_{1}\left(d_{4}\right),\sigma_{3}\left(d_{5}\right)⟶1,\;\sigma_{3}\left(d_{5}\right),\sigma_{3}\left(d_{6}\right)⟶3,\sigma_{3}\left(d_{6}\right),\sigma_{1}\left(d_{7}\right)⟶1,\\ \sigma_{1}\left(d_{7}\right),\sigma_{3}\left(d_{8}\right)⟶1,\;\sigma_{3}\left(d_{8}\right),\sigma_{2}\left(d_{9}\right)⟶2,\sigma_{2}\left(d_{9}\right),\sigma_{2}\left(d_{10}\right)⟶2,\\ \sigma_{2}\left(d_{10}\right),\sigma_{2}\left(d_{11}\right)⟶2,\;\sigma_{3}\left(d_{11}\right),\sigma_{1}\left(d_{12}\right)⟶1,\sigma_{1}\left(d_{12}\right),\sigma_{0}\left(d_{13}\right)⟶0. \end{array}$$

The maximum link dimension is 3, indicating the relationship between the diagnosis classes.

#### 3.3.1. Calculating the Structure Vectors

As mentioned in the definitions, the vector *Q*_*q*_ is a simplification basis, created to eliminate the additional impacts in the equivalent simplex sets. The maximum complex dimension with **α**_%70_=7 is 3. Therefore, the first structure vector based on the output is

(5) $$\begin{array}{c} \begin{array}{ccccc} \mathrm{Dimension} & 3 & 2 & 1 & \left\{0\right\} \end{array}. \end{array}$$

The second structure vector *P* is

(6) $$\begin{array}{c} \begin{array}{ccccc} \mathrm{dimensions} & 3 & 2 & 1 & 0 \end{array},\\ P=\left(\begin{array}{cccc} P_{\dim3} & P_{\dim2} & P_{\dim1} & P_{\dim0} \end{array}\right),\\ P=\left(\begin{array}{cccc} 4 & 7 & 10 & 12 \end{array}\right), \end{array}$$

where *P*_*q*_ is the number simplexes greater than or equal to *q* in the set *K* in which *P* is the number of simplex link repetitions (support indices) in the quadruple design and implementation steps of the cryptography algorithms. Based on the values of these two vectors, it is seen that the relationship between the support indices and the quadruple design and implementation steps of the cryptography algorithms is high. This issue indicates the role of support components in the design and implementation of the cryptography algorithms, which should be considered seriously.

#### 3.3.2. Calculating the Obstruction or Flexibility Vector

***Q***^**∗**^**K** represents the number of structural obstructions for simplex interactions in dimension *k*:

(7) $$\begin{array}{c} Q^{*}=Q-I⟶Q^{*}=\left[\begin{array}{cccc} 1 & 1 & 1 & 1 \end{array}\right]-\left[\begin{array}{cccc} 1 & 1 & 1 & 1 \end{array}\right]⟶Q^{*}=\left[\begin{array}{cccc} 0 & 0 & 0 & 0 \end{array}\right]. \end{array}$$

As can be seen, there is no obstruction in any of the communication levels, indicating that there is a significant relationship between the support components at each equivalence class.

#### 3.3.3. Calculating Irregularity

The value of (ecc′(*σ*)) is calculated using the Chinese method. The results for **α**_%70_=7 are shown in Table 7. The calculated irregularity value shows that the indices *d*_2_ (structure/organization), *d*_5_ (human resources/education), *d*_6_ (research and development), and *d*_8_ (management) affect other indices.

#### 3.3.4. Calculating Complexity

Also, the results of *Q*-analysis can be used to describe structure complexity. According to equations (4)–(9) and for **α** **=** **7**, the complexity measure is

(8) $$\begin{array}{c} Q=\left(\begin{array}{cccc} 1, & 1, & 1, & 1 \end{array}\right),\\ \psi \left(K\right)=2\left[\frac{\left(1+2+3+4\right)}{\left(4*5\right)}\right]=1. \end{array}$$

Since, in the above model, there is no obstruction among the component of the equivalent class, it was expected that the complexity of the support components is not high, and the obtained complexity index of 1 verifies this expectation. The system complexity for different alpha-cuts is shown in Figure 5.

#### 3.3.5. Ranking the Support Components of the Design and Implementation of the Cryptography Algorithms

The results of using *A*-analysis are shown in Table 7. The connection strength of the factors in one group is specified with alpha-cut. Therefore, the support components are grouped in 5 levels. Each level describes the priority and importance of the group in developing the cryptography algorithms. In Figure 6 the ranking pyramid of the support components using *Q*-analysis is shown. To allocate proper resources, the components existing in higher levels of the pyramid (Figure 6) are of higher priority.

#### 3.3.6. Validation of the Results

In this section, the results of the cybernetic model and *Q*-analysis for support components' ranking are compared with the results reported in the global cybersecurity index (GCI) in 2015, 2017, and 2018 presented by ITU [36–39]. The GCI reports are focused on five indices, including “legal cases, organization necessities, technical issues, capacity building, and cooperation,” and the subindices include legal, technical, organization, capacity building, and cooperation. According to the presented indices and subindices, it is clear that the “rules,” “standard,” “research and development,” “education,” and “management” are of higher priority in security establishment. Although our research is more skilled and detailed compared to the GCI reports, but the results verify our findings. Also, Table 8 shows the ranking of the support components obtained using *Q*-analysis.

#### 3.3.7. Executing the Model and Analyzing the Results of the Objectives' Impact on Design Steps of the Cryptography Algorithms' Matrix

In this section, the role of the seven components on the quadruple design and implementation steps of the cryptography algorithm is analyzed with *Q*-analysis. Using the *Q*-analysis method and the 7∗4 matrix obtained from the relationship of the cryptography algorithms' design objectives on their quadruple steps, their indices are ranked.

#### 3.3.8. Calculating the Incidence Matrix and Executing the Model

First, the incidence matrix is obtained for the data matrix shown in Figure 2. It can be seen in Table 9 that each element of the two sets represents which indice. The incidence matrix calculated from the data matrix for *α*_%5_=40 is given in Table 10. The results of implementing the model for *α*_%5_=40 are given in Figure 7.

## 4. Geometric Representation

In the sample with *α*_%5_=40, *d*_*i*_*s* are

(9) $$\begin{array}{c} d_{1}=\left\{c_{1},c_{2},c_{3},c_{4}\right\},\\ d_{2}=\left\{\;\right\},\\ d_{3}=\left\{c_{1},c_{3},c_{4}\right\},\\ d_{4\;}=\left\{c_{3},c_{4}\right\},\\ d_{5\;}=\left\{\;\right\},\\ d_{6\;}=\left\{c_{1},c_{2},c_{3},c_{4}\right\},\\ d_{7\;}=\left\{\;\right\}. \end{array}$$

The simplexes of **σ**_**p**_(**d**_**i**_) are also

(10) $$\begin{array}{c} \sigma_{3}\left(d_{1}\right)\sigma_{-1}\left(d_{2}\right)\sigma_{2}\left(d_{3}\right)\sigma_{1}\left(d_{4}\right)\sigma_{-1}\left(d_{5}\right)\sigma_{3}\left(d_{6}\right)\sigma_{-1}\left(d_{7}\right). \end{array}$$

Therefore, the complex dimension is 3. In other words, the discriminant classes *d*_1_ (security) and *d*_6_ (speed) have the largest dimension.

### 4.1. Calculating the Structure Vectors

As mentioned, the vector *Q*_*q*_ is a simplification basis to eliminate the additional effects in the set of equivalent simplexes. The maximum complex dimension for *α*_%5_=40 is 3. Therefore, the first structure vector based on the output is

(11) $$\begin{array}{c} \begin{array}{ccccc} \mathrm{Dimension} & 3 & 2 & 1 & 1 \end{array},\\ Q=\left(\begin{array}{cccc} 1 & 1 & 1 & 1 \end{array}\right),\\ \begin{array}{ccccc} \mathrm{Dimension} & 3 & 2 & 1 & 0 \end{array},\\ P=\left(\begin{array}{cccc} 2 & 3 & 4 & 7 \end{array}\right). \end{array}$$

The second structure vector *P* is

(12) $$\begin{array}{c} P=\left(\begin{array}{cccc} 2 & 3 & 4 & 7 \end{array}\right). \end{array}$$

### 4.2. Calculating the Obstruction Vector or Inflexibility

**Q**^**∗**^_**K**_ represents the number of structural obstructions for simplex interactions in dimension *k*, which is as follows for *α*_%5_=40:

(13) $$\begin{array}{c} Q^{*}=Q-I⟶Q^{*}=\left[\begin{array}{cccc} 2 & 1 & 1 & 3 \end{array}\right]-\left[\begin{array}{cccc} 1 & 1 & 1 & 1 \end{array}\right]⟶Q^{*}=\left[\begin{array}{cccc} 0 & 0 & 0 & 0 \end{array}\right]. \end{array}$$

According to the obtained values, it can be concluded that there are no structural obstructions among the main design indices of the cryptography algorithms. That is, multiple objectives are considered simultaneously by the cryptography algorithm designers.

### 4.3. Calculating Irregularity

The results of applying the Chinese method (ecc‘(*σ*)) for calculating irregularity for *α*_%5_=40 are shown in Table 11. The calculated irregularity value shows that indices *d*_1_ (security) and *d*_6_ (speed) have received more attention compared to other indices.

### 4.4. Calculating Complexity

Structural complexity for a sample with *α*_%5_=40 is

(14) $$\begin{array}{c} \begin{array}{ccccc} \mathrm{dimensions} & 3 & 2 & 1 & 0, \end{array}\\ Q=\left(\begin{array}{cccc} Q_{\dim3} & Q_{\dim2} & Q_{\dim1} & Q_{\dim0} \end{array}\right),\\ Q=\left(\begin{array}{cccc} 1 & 1 & 1 & 1 \end{array}\right),\\ \psi \left(K\right)=2\left[\frac{\left(1+2+3+4\right)}{\left(4*5\right)}\right]=1. \end{array}$$

Since, in the above model, there was no obstruction among the components of the equivalent classes in any of the communication levels, it was expected that there is not a high complexity among objectives of the cryptography algorithm design; and, the complexity index of 1 verified this expectation. The system complexity for different alpha-cuts is shown in Figure 8. As can be seen, the system complexity is 1 for all significant values of alpha.

### 4.5. Prioritizing the Parameters of the Main Objectives of the Cryptography Algorithm Design Using *Q*-Analysis

According to the analysis results, the parameters can be classified into 5 levels. These levels are shown in Table 12 and Figure 9. Each level indicates a priority and importance of the group in the development of cryptography algorithms. To allocate proper resources, the components at the higher levels of the pyramid are of higher priority. As can be seen, three objectives of security, speed, and optimal usage of resources have the highest priority for the design of cryptography algorithms.

### 4.6. Executing the Model and Analyzing the Results for the Cryptography Algorithm Implementation Techniques

The interaction matrix between the 29 extracted techniques and the seven main objectives is shown in Figure 10. The purpose of this section is to rank the cryptography algorithm implementation techniques to achieve the goals of interest.

### 4.7. Calculating the Incidence Matrix and Executing the Model

The data matrix *A* is comprised of two sets. The set *D* represents the employed techniques, and the set *C* represents the seven main design objectives (Table 13):

(15) $$\begin{array}{c} D=\left\{d_{1},\;d_{2},\;\ldots ,\;d_{29}\right\},\\ C=\left\{c_{1},\;c_{2},\ldots ,c_{7}\right\}. \end{array}$$

Some parts of the incidence matrix calculated from the data matrix A for *α*_%3_ are shown in Table 14, and the results of the *Q*-analysis model for *α*_%3_= 24 are shown in Figure 11.

### 4.8. Geometric Representation

In the sample with **α**_%3_=24, the dis are

(16) $$\begin{array}{c} d_{1}=\left\{c_{1}\right\},\\ d_{2}=\left\{\;\right\},\\ d_{3}=\left\{\;\right\},\\ d_{4}=\left\{\;\right\},\\ d_{5}=\left\{\;\right\},\\ d_{6}=\left\{\;\right\},\\ d_{7}=\left\{\;\right\},\\ d_{8}=\left\{\;\right\},\\ d_{9}=\left\{\;\right\},\\ d_{10}=\left\{\;\right\},\\ d_{11}=\left\{c_{1}\right\},\\ d_{12}=\left\{\;\right\},\\ d_{13}=\left\{c_{5}\right\},\\ d_{14}=\left\{\;\right\},\\ d_{15}=\left\{c_{1},c_{4},c_{5}\right\},\\ d_{16}=\left\{\;\right\},\\ d_{17}=\left\{\;\right\},\\ d_{18}=\left\{\;\right\},\\ d_{19}=\left\{c_{1}\right\},\\ d_{20}=\left\{\;\right\},\\ d_{21}=\left\{\;\right\},\\ d_{22}=\left\{c_{3}\right\},\\ d_{23}=\left\{\;\right\},\\ d_{24}=\left\{\;\right\},\\ d_{25}=\left\{\;\right\},\\ d_{26}=\left\{\;\right\},\\ d_{27}=\left\{c_{1}\right\},\\ d_{28}=\left\{\;\right\},\\ d_{29}=\left\{\;\right\}. \end{array}$$

The simplexes of **σ**_**p**_(**d**_**i**_) are

(17) $$\begin{array}{c} \sigma_{0}\left(d_{1}\right),\\ \sigma_{-1}\left(d_{2}\right),\\ \sigma_{-1}\left(d_{3}\right),\\ \sigma_{-1}\left(d_{4}\right),\\ \sigma_{-1}\left(d_{5}\right),\\ \sigma_{-1}\left(d_{6}\right),\\ \sigma_{-1}\left(d_{7}\right),\\ \sigma_{-1}\left(d_{8}\right),\\ \sigma_{-1}\left(d_{9}\right),\\ \sigma_{-1}\left(d_{10}\right),\\ \sigma_{0}\left(d_{11}\right),\\ \sigma_{-1}\left(d_{12}\right),\\ \sigma_{0}\left(d_{13}\right),\\ \sigma_{-1}\left(d_{14}\right),\\ \sigma_{2}\left(d_{15}\right),\\ \sigma_{-1}\left(d_{16}\right),\\ \sigma_{-1}\left(d_{17}\right),\\ \sigma_{-1}\left(d_{18}\right),\\ \sigma_{0}\left(d_{19}\right),\\ \sigma_{-1}\left(d_{20}\right),\\ \sigma_{-1}\left(d_{21}\right),\\ \sigma_{0}\left(d_{22}\right),\\ \sigma_{-1}\left(d_{23}\right),\\ \sigma_{-1}\left(d_{24}\right),\\ \sigma_{-1}\left(d_{25}\right),\\ \sigma_{-1}\left(d_{26}\right),\\ \sigma_{0}\left(d_{27}\right),\\ \sigma_{-1}\left(d_{28}\right),\\ \sigma_{-1}\left(d_{29}\right). \end{array}$$

Therefore, the complex dimension is 2. In other words, the discriminant class *d*_15_ (basic sciences) has the largest dimension.

### 4.9. Calculating the Dimensions and the *Q*-Link

In the alpha defined for cryptography algorithm implementation techniques to achieve the defined goals, the obtained *q*-link shows that these techniques are relatively independent although there is a weak relationship between some techniques. *Q*-link in the samples with *α*_%3_=24 between each two subsequent *d*_i_ is as follows:

(18) $$\begin{array}{c} \sigma_{0}\left(d_{1}\right),\sigma_{-1}\left(d_{2}\right)⟶-1,\\ \sigma_{-1}\left(d_{2}\right),\sigma_{-1}\left(d_{3}\right)⟶-1,\\ \sigma_{0}\left(d_{3}\right),\sigma_{-1}\left(d_{4}\right)⟶-1,\\ \sigma_{-1}\left(d_{4}\right),\sigma_{-1}\left(d_{5}\right)⟶-1,\\ \sigma_{-1}\left(d_{5}\right),\sigma_{-1}\left(d_{6}\right)⟶-1,\\ \sigma_{-1}\left(d_{6}\right),\sigma_{-1}\left(d_{7}\right)⟶-1,\\ \sigma_{-1}\left(d_{7}\right),\sigma_{-1}\left(d_{8}\right)⟶-1,\\ \sigma_{-1}\left(d_{8}\right),\sigma_{-1}\left(d_{9}\right)⟶-1,\\ \sigma_{-1}\left(d_{9}\right),\sigma_{-1}\left(d_{10}\right)⟶-1,\\ \sigma_{-1}\left(d_{10}\right),\sigma_{0}\left(d_{11}\right)⟶-1,\\ \sigma_{0}\left(d_{11}\right),\sigma_{-1}\left(d_{12}\right)⟶-1,\\ \sigma_{-1}\left(d_{12}\right),\sigma_{0}\left(d_{13}\right)⟶-1,\\ \sigma_{0}\left(d_{13}\right),\sigma_{-1}\left(d_{14}\right)⟶-1,\\ \sigma_{-1}\left(d_{14}\right),\sigma_{2}\left(d_{15}\right)⟶-1,\\ \sigma_{2}\left(d_{15}\right),\sigma_{-1}\left(d_{16}\right)⟶-1,\\ \sigma_{-1}\left(d_{16}\right),\sigma_{-1}\left(d_{17}\right)⟶-1,\\ \sigma_{-1}\left(d_{17}\right),\sigma_{-1}\left(d_{18}\right)⟶-1,\\ \sigma_{-1}\left(d_{18}\right),\sigma_{0}\left(d_{19}\right)⟶-1,\\ \sigma_{0}\left(d_{19}\right),\sigma_{-1}\left(d_{20}\right)⟶-1,\\ \sigma_{-1}\left(d_{20}\right),\sigma_{-1}\left(d_{21}\right)⟶-1,\\ \sigma_{-1}\left(d_{21}\right),\sigma_{0}\left(d_{22}\right)⟶-1,\\ \sigma_{0}\left(d_{22}\right),\sigma_{-1}\left(d_{23}\right)⟶-1,\\ \sigma_{-1}\left(d_{23}\right),\sigma_{-1}\left(d_{24}\right)⟶-1,\\ \sigma_{-1}\left(d_{24}\right),\sigma_{-1}\left(d_{25}\right)⟶-1,\\ \sigma_{-1}\left(d_{25}\right),\sigma_{-1}\left(d_{26}\right)⟶-1,\\ \sigma_{-1}\left(d_{26}\right),\sigma_{0}\left(d_{27}\right)⟶-1,\\ \sigma_{0}\left(d_{27}\right),\sigma_{-1}\left(d_{28}\right)⟶-1,\\ \sigma_{-1}\left(d_{28}\right),\sigma_{-1}\left(d_{29}\right)⟶-1. \end{array}$$

### 4.10. Calculating the Structure Vectors

Therefore, the first structure vector based on the software output is

(19) $$\begin{array}{c} Q=\left(\begin{array}{ccc} 1 & 1 & 2 \end{array}\right). \end{array}$$

The second structure vector *P* is

(20) $$\begin{array}{c} P=\left(\begin{array}{ccc} 1 & 1 & 29 \end{array}\right). \end{array}$$

Since the large values of *P* of higher dimensions demonstrate more links, the second structure vector calculated for the alpha of interest shows that the relationship between the cryptography algorithm implementation techniques is minimum.

### 4.11. Calculating the Obstruction or Inflexibility Vector

The obstruction vector (**Q**^**∗**^) for a sample with *α*_%3_=24 is

(21) $$\begin{array}{c} Q^{*}=Q-I⟶Q^{*}=\left[\begin{array}{ccc} 1 & 1 & 2 \end{array}\right]-\left[\begin{array}{ccc} 1 & 1 & 1 \end{array}\right]⟶Q^{*}=\left[\begin{array}{ccc} 0 & 0 & 1 \end{array}\right].\; \end{array}$$

The value of **Q**^**∗**^_**K**_ represents the number of structural limitations or obstructions for the cryptography techniques' interaction at dimension *k*. As can be seen from the calculated obstruction vector, there is a significant relationship at some levels.

### 4.12. Calculating Irregularity

Irregularity is the integration degree of a cryptography method in the total complex. Measuring irregularity (ecc') for *α*_%3_=24 is shown in Table 15. As can be seen, irregularity for the discriminant class *d*_15_ indicates that this technique is isolated from other techniques.

### 4.13. Calculating Complexity

Structure complexity for a sample with *α*_%3_=24 is

(22) $$\begin{array}{c} Q=\left(\begin{array}{ccc} 1 & 1 & 2 \end{array}\right),\\ \psi \left(K\right)=2\left[\frac{\left(2+2+3\right)}{\left(3*4\right)}\right]=1.17. \end{array}$$

The system complexity for different values of alpha is shown in Figure 12. As can be seen, the total complexity of the system for large values alpha tends to stability.

### 4.14. Ranking the Cryptography Algorithm Implementation Techniques

These techniques can be classified into 5 levels using the analysis of the obtained results. These levels can be seen in Table 16 and Figure 13. The link power of the factors in one group is specified with alpha. Each level describes priority and importance of the group in the development of cryptography algorithms. Accordingly, six methods of basic science, key management, using hardware methods, using steganography, Avalanche effect, and using hybrid method are the most important cryptography algorithm implementation techniques to achieve the main objectives.

## 5. Conclusion

In this study, the design and implementation model of the cryptography algorithms is designed in three levels and its effective components are extracted. To organize the components, in addition to elimination of the additional components through the measure reduction algorithm, a proper classification is applied to examine the mutual effects. After classification, three 13 ∗ 4, 7 ∗ 4, and 29 ∗ 7 matrices are constituted, and the model is implemented on these three matrices. To implement the designed model, *Q*-analysis is used. Accordingly, for support indices, five indices of high priority include human resources, research and development, management, organization/structure, and equipment. For the algorithm design objectives index, five high priority indices include security, speed, optimal usage of resources, and simplicity. For the indices related to implementation techniques of the cryptography algorithms, the most applied techniques for achieving the determined objectives include using basic science, hardware and software methods, using key management, hybrid method, steganography, Avalanche effect, and using artificial intelligence. In the future work, we will consider the following cases.

A plan should be formulated according to the priorities. According to the outputs of this study and the presented priorities, the following topics can be investigated in future studies:

1. Presenting a comprehensive model for generating various cryptography algorithms based on the priorities of interest
2. Examining and formulating a model about the role of basic science for design and implementation of cryptography algorithms considering the significant role of “basic science” in implementation of the cryptography algorithms and about the role of schools and universities
3. Presenting a model for design and implementation of cryptography algorithms in the IoT infrastructure with optimal resource usage

## Figures and Tables

**Figure 1:** Main process of design and implementation of cipher algorithms at the highest level.

**Figure 2:** General schematic of the conceptual model of the cipher algorithm design.

**Figure 3:** The cybernetic model of design and implementation of cipher algorithms at level 3.

**Figure 4:** Implementation results of the model for support components of the cryptography algorithms' design with *α*=%70.

**Figure 5:** System complexity of the support indices of design and implementation of the cryptography algorithms for different alpha-cuts.

**Figure 6:** The ranking pyramid of the support components using *Q*-analysis.

**Figure 7:** The results of executing the model for design objectives' indices with *α* = 40.

**Figure 8:** System complexity of the cryptography algorithm design objectives for different alpha-cuts.

**Figure 9:** Prioritizing the design and implementation objectives of the cryptography algorithms using *Q*-analysis.

**Figure 10:** Prioritizing the design and implementation objectives of the cryptography algorithms using *Q*-analysis.

**Figure 11:** Results of executing the model for cryptography algorithm implementation techniques with *α*_%3_=24.

**Figure 12:** System complexity of cryptography algorithm implementation techniques for different alpha-cuts.

**Figure 13:** Prioritizing the implementation techniques of the cryptography algorithms using *Q*-analysis.

**Table 1:** The importance of information security needs in telemedicine technology in the field of information transmission.

Data transfer	Very important	Important	No idea	Nonsignificant
Implement network protocols to ensure the transmission of information and check its integrity	2/65%	4/30%	4/3	0
Establish a communication protocol to share information between local health institutions	50%	37%	13	0
Encrypt important files and information	2/62%	6/35%	0	2/2
Investigation of encryption mechanism by technical team of security assessor	5/56%	3/28%	15/2	0
Use combinations of numbers and letters for encryption	2/68	25	6/8	0
Use uppercase and lowercase letters for encryption to access remote network networks	50%	24%	17/4	8/7
Methods for controlling the integrity of application information	3/53%	6/35%	8/9	2/2

**Table 2:** The 13-component interaction matrix of the support and the main design and implementation processes of cryptography algorithms.

			Main process				Level 1
			Cryptography algorithms				Level 2
			Application	Theoretical basis	Implementation	Evaluation	Level 3
Support process	Software	Culture	5	6	5	2	.
		Organization/structure	8	7	7	7	.
		International and public relations	5	4	4	7	.
		Financial resources	7	6	7	6	.
		Human resources and education	8	10	10	9	.
		Research and development	10	8	8	10	.
		Rules	7	4	5	10	.
		Management	9	7	8	7	.
		FAVA	10	5	8	7	.
		Standard	10	3	8	10	.
	Hardware	Equipment	8	6	7	8	
		Infrastructure	9	5	5	7	
		Material	7	2	5	5	

**Table 3:** The relationship matrix of the objectives with the design process of the cryptography algorithms.

Main process objectives	Application	Theoretical basis	Implementation	Evaluation
Security	203	386	516	516
Simplicity	5	23	38	38
Resources	41	30	81	81
Flexibility	15	28	45	45
Scalability	6	11	22	22
Speed	72	146	247	247
Reliability	2	10	11	11

**Table 4:** A part of the interaction matrix between the cryptography algorithm implementation techniques and the seven objectives.

Level 3		Security	Simplicity	Using resources	Flexibility	Scalability	Speed	Reliability
**Support process**	Avalanche effect	**32**	**0**	**0**	**0**	**0**	**0**	**0**
	Digital signature	**1**	**0**	**0**	**0**	**0**	**0**	**0**
	Block size	**1**	**1**	**0**	**0**	**2**	**0**	**0**
	Image sharing	**0**	**0**	**0**	**1**	**0**	**0**	**0**
	Parallel processing	**0**	**0**	**0**	**1**	**12**	**0**	**0**
	Threshold technique	**3**	**1**	**0**	**0**	**0**	**0**	**0**
	Data mining	**1**	**0**	**0**	**0**	**0**	**0**	**0**
	Binary tree	**1**	**0**	**0**	**0**	**3**	**0**	**0**
	Cycle	**5**	**2**	**0**	**0**	**12**	**0**	**0**
	Multistage crypto	**1**	**0**	**0**	**0**	**0**	**0**	**0**
	Hybrid method	**30**	**3**	**0**	**2**	**9**	**0**	**2**
	Hardware	**0**	**0**	**7**	**0**	**0**	**0**	**0**

**Table 5:** Sets of *d*_*i*_*s* and *c*_*i*_*s*; support indices based on the data matrix.

*d*_1_	Culture
*d*_2_	Structure/organization
*d*_3_	International/public relations
*d*_4_	Financial
*d*_5_	Human resources/education
*d*_6_	Research and development
*d*_7_	Rules
*d*_8_	Management
*d*_9_	FAVA
*d*_10_	Standard
*d*_11_	Equipment
*d*_12_	Infrastructure
*d*_13_	Material
*C*_1_	Application
*C*_2_	Theoretical basis
*C*_3_	Implementation
*C*_4_	Evaluation

**Table 6:** The incidence matrix of the support indices' impact of the design steps of the cryptography algorithms with *α*=%70.

	*C*_1_	*C*_2_	*C*_3_	*C*_4_
*d*_1_	0	0	0	0
*d*_2_	1	1	1	1
*d*_3_	0	0	0	1
*d*_4_	1	0	1	0
*d*_5_	1	1	1	1
*d*_6_	1	1	1	1
*d*_7_	1	0	0	1
*d*_8_	1	1	1	1
*d*_9_	1	0	1	1
*d*_10_	1	0	1	1
*d*_11_	1	0	1	1
*d*_12_	1	0	0	1
*d*_13_	1	0	0	0

**Table 7:** The irregularity of the data matrix parameters for **α** **=** **7**.

**σ**	**q**_**i**_	∑**q**_**i**_/**σ**_**i**_	**q**_**max**_	**ecc**′(**σ**)=2∑**q**_**i**_/**σ**_**i**_/**q**_**max**_(**q**_**max**_+1)
**d**_2_, **d**_5_, **d**_6_, **d**_8_	*q*_*i*_=3,2,1	3.64	3	0.61
**d**_9_, **d**_10_, **d**_11_	*q*_*i*_=2,1	0.64	3	0.11
**d**_4_, **d**_7_, **d**_12_	*q*_*i*_=1	0.14	3	0.02

**Table 8:** Ranking of the support components using *Q*-analysis.

Relationship of the support components with the design and implementation of the cryptography algorithms (*q* = 0)	
No relationship: *α*=0%; complete relationship: *α*=100%	
Human resource, R&D, rules, FAVA, and standard	*α*_%100_= 10
Management and infrastructure	*α*_%90_= 9
Organization/structure and equipment	*α*_%80_= 8
International and public relations, financial resources, and material	*α*_%70_= 7
Culture	*α*_%60_= 6
All components	*α*_%60_= 5

**Table 9:** Set of d_i_s and c_i_s; the objectives' indices.

Theoretical basis	*C*_2_	Reliability	*d*_7_	Scalability	*d*_5_	Resources	*d*_3_	Security	*d*_1_
Implementation	*C*_3_	Application	*C*_1_	Speed	*d*_6_	Flexibility	*d*_4_	Simplicity	*d*_2_
Evaluation	*C*_4_								

**Table 10:** The incidence matrix of the design objectives of the cryptography algorithms with **α** **=** **40**.

	*c*_1_	*c*_2_	*c*_3_	*c*_4_
*d*_1_	1	1	1	1
*d*_2_	0	0	0	0
*d*_3_	1	0	1	1
*d*_4_	0	0	1	1
*d*_5_	0	0	0	0
*d*_6_	1	1	1	1
*d*_7_	0	0	0	0

**Table 11:** Irregularity of the cryptography objectives' parameters in the data matrix *A* for *α*_%5_.

*σ*	*q*_*i*_	∑*q*_*i*_/*σ*_*i*_	*q*_max_	ecc′(*σ*)=2∑*q*_*i*_/*σ*_*i*_/*q*_max_(*q*_max_+1)
*d*_1_ and *d*_6_	*q*_*i*_=3,2, and 1	4.33	3	0.72
*d*_3_	*q*_*i*_=2 and 1	1.33	3	0.26
*d*_4_	*q*_*i*_=1	0.33	3	0.06

**Table 12:** Ranking the objectives' parameters considering different cuts in *Q*-analysis.

The equivalence class for the parameters with minimum relation level (*q* = 0)	*α*
Security	*α*_%50_= 244
Speed	*α*_%30_= 244
Resources	*α*_%15_= 122
Flexibility	*α*_%5_= 40
Simplicity-scalability	*α*_%2_= 16
(All parameters)	?

**Table 13:** Set of dis and cis; the techniques employed for implementing cryptography algorithms.

Flexibility	*C*_4_	Fuzzy logic	*d*_25_	Storage space	*d*_17_	Cycle	*d*_9_	Avalanche effect	*d*_1_
Scalability	*C*_5_	Software	*d*_26_	Clustering	*d*_18_	Multiple step	*d*_10_	Digital signature	*d*_2_
Speed	*C*_6_	Steganography	*d*_27_	Key	*d*_19_	Hybrid method	*d*_11_	Block size	*d*_3_
Reliability	*C*_7_	Music harmony	*d*_28_	Graph	*d*_20_	Hardware	*d*_12_	Image sharing	*d*_4_
		Artificial intelligence	*d*_29_	Characteristic oriented	*d*_21_	Hardware	*d*_13_	Parallel processing	*d*_5_
		Security	*C*_1_	Energy consumption	*d*_22_	Occupation area	*d*_14_	Threshold technique	*d*_6_
		Simplicity	*C*_2_	Bandwidth consumption	*d*_23_	Basic science	*d*_15_	Data mining	*d*_7_
		Resources	*C*_3_	Memory consumption	*d*_24_	Compression	*d*_16_	Binary tree	*d*_8_

**Table 14:** The incidence matrix of the cryptography algorithm implementation techniques with *α* = 24.

	*C*_1_	*C*_2_	*C*_3_	*C*_4_	*C*_5_	*C*_6_	*C*_7_
*d*_1_	1	0	0	0	0	0	0
*d*_2_	0	0	0	0	0	0	0
*d*_3_	0	0	0	0	0	0	0
*d*_4_	0	0	0	0	0	0	0
*d*_5_	0	0	0	0	0	0	0
*d*_6_	0	0	0	0	0	0	0
*d*_7_	0	0	0	0	0	0	0
*d*_8_	0	0	0	0	0	0	0
*d*_9_	0	0	0	0	0	0	0
*d*_10_	0	0	0	0	0	0	0
*d*_11_	1	0	0	0	0	0	0
*d*_12_	0	0	0	0	0	0	0

**Table 15:** Irregularity of the cryptography algorithm implementation techniques for *α*_%3_=24.

**σ**	**q**_**i**_	∑**q**_**i**_/**σ**_**i**_	**q**_**max**_	**ecc**′(**σ**)=2∑**q**_**i**_/**σ**_**i**_/**q**_**max**_(**q**_**max**_+1)
**d**_15_	*q*_*i*_=2,1	3	2	1
-	*q*_*i*_=1	1	2	0.33

**Table 16:** Ranking the implementation techniques of the cryptography algorithms considering various alpha-cuts using *Q*-analysis.

Equivalence classes for the parameters with minimum relationship level (*q* = 0)	*α*
Basic sciences	*α*_%20_= 163
Key	*α*_%10_= 81
Hardware and steganography	*α*_%5_= 40
Avalanche effect and hybrid method	*α*_%3_= 24
{Artificial intelligence, software}, {occupation area, energy consumption, memory consumption}	*α*_%2_= 16

## Data Availability

The data used to support the findings of the study are available from the corresponding author upon request.
